# Effect of Xuefu Zhuyu Capsule on Myocardial Infarction: Network Pharmacology and Experimental Verification

**DOI:** 10.1155/2023/5652276

**Published:** 2023-01-31

**Authors:** Jinlong Duan, Jianguo Lin, Nixue Zhang, Qingqing Wang, Na Li, Kuiwu Yao

**Affiliations:** ^1^Guang'anmen Hospital, China Academy of Chinese Medical Sciences, Beijing, China; ^2^Tianjin University of Traditional Chinese Medicine, Tianjin, China; ^3^Institute of Chinese Materia Medica, China Academy of Chinese Medical Sciences, Beijing, China; ^4^Beijing University of Chinese Medicine, Beijing, China; ^5^Eye Hospital, China Academy of Chinese Medical Sciences, Beijing, China

## Abstract

**Background:**

Myocardial infarction (MI) is the most severe manifestation of cardiovascular disease. Xuefu Zhuyu Capsule (XFC), a proprietary Chinese medicine, is widely used in various cardiovascular diseases. At present, the molecular mechanism of XFC remains unclear.

**Objective:**

To explore the mechanism of anti-MI effects of XFC by combining network pharmacology and experiments.

**Methods:**

TCMSP, GeneCards, and DisGeNET databases were used to find the target of XFC. PPI analysis was performed by the STRING database. KEGG and GO analyses were performed by Metascape Database. Molecular docking was performed by Autodock Vina. HE staining, echocardiography, immunofluorescence, and TUNEL were performed to verify the prediction results.

**Results:**

Network pharmacology showed that quercetin, kaempferol, *β*-sitosterol, luteolin, and baicalein were the main active ingredients of XFC. TNF, IL6, TP53, VEGFA, JUN, CASP3, and SIRT1 were the main targets of XFC. KEGG results showed that key genes were mainly enriched in lipid and atherosclerosis, PI3K-Akt signaling pathway, MAPK signaling pathway, and NF-*κ*B signaling pathway. HE staining showed that XFC could improve the morphology of myocardial tissue. Echocardiography showed that XFC could improve cardiac function. TUNEL showed that XFC could reduce cardiomyocyte apoptosis. Immunofluorescence showed that XFC could reduce the expression of *α*-smooth muscle actin (*α*-SMA) and increase the expression of CD31. In addition, we found that XFC may exert its therapeutic effects through SIRT1.

**Conclusion:**

This study demonstrated that SIRT1 may be the target of XFC in the treatment of MI. The active ingredients of XFC and SIRT1 can be stably bound. XFC could inhibit apoptosis, promote angiogenesis, and improve myocardial fibrosis through SIRT1.

## 1. Introduction

Myocardial infarction (MI) is the most severe manifestation of cardiovascular disease (CVD), which affects more than 7 million individuals worldwide each year [1]. The usual initiating mechanism for MI is the rupture or erosion of a vulnerable, lipid-laden, atherosclerotic coronary plaque, resulting in exposure of circulating blood to a highly thrombogenic core and matrix materials in the plaque [2]. The method of saving ischemic myocardium from MI is timely reperfusion, including drug thrombolysis and percutaneous coronary intervention; however, the process of reperfusion may lead to arrhythmia, myocardial stunning, microvascular obstruction, and lethal myocardial reperfusion injury [3, 4].

Traditional Chinese medicine (TCM) has a long history of treating MI. Our research group has previously found that blood-activating Chinese herbal medicine has an improving effect on ischemic heart disease [5–7]. Xuefu Zhuyu Capsule (XFC) is a TCM formula that originated from the Qing Dynasty, which has the function of promoting blood circulation, removing blood stasis, moving Qi, and relieving pain, and is widely used in various CVD [8–10]. XFC is composed of 11 types of herbs, including *Semen Persicae, Flos Carthami, Radix Rehmanniae, Radix Angelicae sinensis, Radix Achyranthis Bidentatae, Radix Platycodi, Radix chuanxiong, Radix Paeoniae Rubra, Fructus Aurantii, Radix Glycyrrhizae, Radix Bupleuri.* Currently, the active ingredients from XFC have been shown to have anti-inflammatory, antioxidative, antiapoptotic, and autophagy-modulating effects, however, the mechanism of XFC in improving MI has not been clarified [6, 11, 12].

Network pharmacology is a new subject based on systems biology and bioinformatics, which can elucidate the mechanism of drug action at the molecular level [13, 14]. The comprehensive and systematic concept of network pharmacology accords with the characteristics of multicomponent, multitarget, and multipathway of TCM. Therefore, in this study, we aimed to explore the active ingredients, therapeutic targets, and signaling pathways of XFC in the treatment of MI through network pharmacology and *in vivo*. Our study may provide evidence for the pharmacological effects of Chinese herbal compounds on MI. A flowchart of the study approach is shown in Figure 1.

## 2. Materials and Methods

### 2.1. Network Pharmacology Analysis

#### 2.1.1. XFC Targets and MI Targets

Ingredients of each herb in XFC were obtained from Traditional Chinese Medicine Systems Pharmacology Database and Analysis Platform (TCMSP, https://tcmspw.com) [15], the TCMSP parameter was set as bioavailability (OB) ≥30% and drug-like properties (DL) ≥0.18, as suggested by the TCMSP. Disease targets of MI were collected by the GeneCards database (https://www.genecards.org/) [16] and the DisGeNET database (https://www.disgenet.org/) [17]. The verified and predictive targets of XFC to treat MI were obtained by overlapping these targets.

#### 2.1.2. Protein-Protein Interaction (PPI) and Gene Enrichment Analysis

PPI analysis of overlapping targets was performed using the STRING platform [18], and the calculation results were imported into Cytoscape 3.9.0 software [19] for network topology analysis. Screen for key targets using the CytoHubba plugin. Gene enrichment analysis of overlapping targets was performed through the Metascape database [20]. It mainly includes molecular function (MF), cellular components (CC), and biological process (BP), KEGG. The parameters of the Metascape database were set as follows: min overlap: 3, *P* value cutoff: 0.01, and min enrichment: 1.5. Hiplot (https://hiplot-academic.com/) [21] is used to visualize the results.

#### 2.1.3. Molecular Docking

Key targets and active ingredients were selected for molecular docking. The key target structure was obtained through the PDB database (https://www.rcsb.org/), and the key active ingredients structure was obtained through the PubChem database (https://pubchem.ncbi.nlm.nih.gov/). PyMOL, Autodock Vina [22], and PLIP (https://plip-tool.biotec.tu-dresden.de/) [23] were used to conduct molecular docking.

### 2.2. Experimental Validation

#### 2.2.1. Drug and Animals

XFC was purchased from Tianjin Hongrentang Pharmaceutical Co., Ltd. (Approval number: Z12020223). EX527 was purchased from Selleckchem, USA, Product No: S1541, male Wistar rats (weighing 190–210 g), purchased from Huafukang Biotechnology Co., Ltd. (Beijing, China). All rats were housed in specific pathogen-free animal rooms in the laboratory animal center of Guang'anmen hospital, China Academy of Chinese Medical Sciences. The temperature of the animal room is 20–25°C, and the relative humidity is 55–60%; all rat feeding methods and animal experiment procedures strictly follow the relevant guidelines stipulated by the experimental animal ethics committee of Guang' anmen Hospital, China Academy of Chinese Medical Sciences.

#### 2.2.2. Model of MI and Drug Treatment

The rats' model of MI was established by left anterior descending (LAD) ligation as previously described [24]. Rats were anesthetized with pentobarbital sodium (60 mg/kg, i.p.). An incision was made between the 4th and 5th intercostal space on the left side of the rat, the thoracic cavity was opened, the pericardium was torn, and the thorax was gently pressed to squeeze out the heart. Find the left atrial appendage and determine the ligation position (2 mm below the junction of the pulmonary conus and the left atrial appendage). The LAD was ligated at the ligation site, the heart was immediately put back into the thoracic cavity, the incision was closed, and the skin was sutured. Animals in the sham group were only threaded without ligation. An electrocardiograph was performed immediately after modeling, and the ST-Segment elevation was the standard screening model and the rats without ECG changes were excluded. After the operation, the surviving rats were randomly divided into the following four groups: (1) sham-operated group (without LAD ligation); (2) model group (LAD ligation); (3) XFC treated group (LAD ligation and intragastrically administered XFC at 0.432 g/kg [25]); (4) EX527 (SIRT1 inhibitor) group (LAD ligation, intragastrically administered XFC at 0.432 g/kg and intraperitoneal injection of EX527 at 5 mg/kg) [26]. The sham group and model group were given equivalent distilled water. All groups began drug intervention within 12 hours after modeling. The drugs were administered once a day for 4 weeks.

#### 2.2.3. Echocardiographic Evaluation of Cardiac Function

After 4 weeks of administration, the Vevo 3100 Imaging System (Fujifilm Visual Sonics Vevo 3100, Toronto, Canada) was used to observe and record the echocardiographic of rats. After the rats were anesthetized with isoflurane, the rats were fixed in a supine position, and the skin was prepared in front of the left chest. The RMV-716 high-frequency probe was used to take the short axis of the left ventricle, and the level of the mitral valve of the rat heart was detected. The average value of 3 consecutive cardiac cycles was taken for each group. Ultrasound detection indexes: left ventricular short-axis ratio (FS) and left ventricular ejection fraction (EF).

#### 2.2.4. Histological Analysis

After echocardiography, the rats were euthanized, anesthetized by intraperitoneal injection of 1% pentobarbital, fixed in the supine position, quickly opened the chest, and the hearts were removed. Some samples were transferred to a refrigerator at −80°C. Another portion of the sample was fixed with 4% paraformaldehyde and used for subsequent studies. Hematoxylin-eosin (HE) staining was prepared according to standard procedures. The rat heart tissue was fixed, dehydrated, embedded in paraffin, and sliced along the longitudinal axis with a thickness of 4 *μ*m. After HE staining (Beyotime, China), the morphology of cardiac tissue cells was observed under the microscope.

#### 2.2.5. Immunofluorescence Staining

Immunofluorescence staining of CD31, *α*-smooth muscle actin (*α*-SMA), and c-TnI was performed. Briefly, the procedure was as follows: sections were prepared, washed 3 times with PBS, repaired with citrate buffer, washed 3 times with PBS, blocked with sheep embryo serum at 37°C for 15 min, washed 3 times with PBS, incubated with primary antibody at 4°C for 17 h, washed 3 times with PBS, incubated with fluorescently labeled secondary antibody at 37°C for 30 min, washed 3 times with PBS, sealed with DAPI, and photographed with the confocal microscope. Ten fields were randomly selected. Image J software was used to measure the integrated option density (IOD) value of the stained positive part in the captured Image, and the arithmetic mean was taken as the IOD value of the section.

#### 2.2.6. TUNEL Assay

Cardiomyocyte apoptosis was detected by the In Situ Cell Death Detection Kit (11684817910, Roche, Switzerland) according to the manufacturer's protocol. Briefly, the procedure was as follows: paraffin section, dewaxing, hydration, cell permeation, adding TUNEL reaction solution, adding converter-POD, reaction with substrate DAB, counting, and photographing (FV1000, Olympus, Japan). Finally, use Image J software to analyze the pictures, calculate the number of positive cells and total cells in each picture, calculate the percentage of apoptosis, and make a statistical analysis.

### 2.3. Statistical Analysis

Statistical analysis was performed using GraphPad Prism 8. All data are presented as the mean ± standard deviation (SD). One-way analysis of variance followed by Tukey's test was used for multiple comparisons among groups. *P*  <  0.05 was considered statistically significant.

## 3. Results

### 3.1. Network Pharmacologic Prediction Analysis of XFC for MI

#### 3.1.1. Analysis of Drug and Disease Targets

A total of 152 active ingredients and 253 targets corresponding to the active ingredients were collected and 2345 disease targets were collected. The list of the top 20 active ingredients was drawn according to OB values (Table 1). The intersection of drug targets and disease targets was calculated, and 147 overlapping targets were obtained (Figure 2(a)). The ingredients-target network figure (Figure 2(b)) was drawn by active ingredients and targets. From this figure, it can be seen that quercetin, kaempferol, *β*-sitosterol, luteolin, baicalein, stigmasterol, naringenin, isorhamnetin, wogonin, and nobiletin correspond to many targets with large degree values. It is speculated that XFC treatment of MI is mainly these active ingredients with large degree values.

#### 3.1.2. Gene Enrichment Analysis of XFC against MI

PPI processing was conducted on the overlapping targets through the STRING platform, and Cytoscape was used for network topology analysis (Figure 3). The key targets were TNF, IL6, TP53, VEGFA, JUN, CASP3, PTGS2, MAPK3, EGFR, STAT3, and SIRT1. Gene enrichment analysis was conducted on the overlapping targets through the Metascape database. KEGG results showed that key genes were mainly enriched in lipid and atherosclerosis, PI3K-Akt signaling pathway, MAPK signaling pathway, NF-*κ*B signaling pathway, cAMP signaling pathway, and calcium signaling pathway (Figure 4(a)); CC results showed that key genes were mainly enriched in membrane raft, transcription regulator complex, vesicle lumen, receptor complex, and integral component of presynaptic membrane (Figure 4(b)). BP results showed that key genes were mainly enriched in the cellular response to nitrogen compound, response to an inorganic substance, response to the hormone, response to xenobiotic stimulus, and cellular response to lipid (Figure 4(c)). MF results showed that key genes were mainly enriched in DNA-binding transcription factor binding, oxidoreductase activity, kinase binding, protein homodimerization activity, and phosphatase binding (Figure 4(d)). Based on our previous studies and network pharmacology results [12, 27], we selected SIRT1 as the validation gene among these targets.

#### 3.1.3. Molecular Docking Verification

Quercetin, kaempferol, *β*-sitosterol, luteolin, and baicalein were selected as binding ligands, and SIRT1 was selected as the target protein. Molecular docking was performed by Autodock Vina. The results showed that the docking energy was ≤−7 kcal·mol^−1^. It can be seen from Figure 5 that the ligands are stably combined in the binding pocket to form a stable structure. For example, quercetin could bind to the SIRT1 via putative hydrogen bonds to the Arg303, Ser370, Leu372, Lys375, Lys377, and Lys408 residues of SIRT1.

### 3.2. Experimental Verification of XFC against MI

#### 3.2.1. Cardiac Function

The results showed that compared with the sham group, the EF and FS in the model group were significantly decreased (*P* < 0.01). Compared with the model group, the EF and FS in the XFC group were significantly increased (*P* < 0.01), and the EF and FS in the EX527 group showed an upward trend, but there was no statistical significance. Compared with the XFC group, the EF and FS in the EX527 group were significantly decreased (*P* < 0.01) (Figure 6).

#### 3.2.2. Pathological Changes in Heart Tissue

Cardiac pathology was compared by HE staining. The results showed that in the sham group, the myocardial fibers were striated, the nucleus of the myocardial cells was in the middle, and the interstitial blood vessels of the myocardial fibers were normal, without interstitial edema and inflammatory cell infiltration. In the model group, the myocardial space of the ischemic heart was enlarged, the fiber arrangement was disordered, and a large number of inflammatory cells infiltrated. The changes in the XFC group and the EX527 group were between the sham group and the model group, and the degree increased in turn (Figure 7(a)).

#### 3.2.3. Changes in Cardiomyocyte Apoptosis

TUNEL assay detects cardiomyocyte apoptosis. The results showed that compared with the sham group, the apoptotic rate of cardiomyocytes in the model group was significantly increased (*P* < 0.01); compared with the model group, the apoptosis rate of cardiomyocytes in the XFC group was significantly decreased (*P* < 0.01). Compared with the XFC group, the apoptosis rate of cardiomyocytes in the EX527 group was significantly increased (*P* < 0.01) (Figure 7(b)).

#### 3.2.4. Changes in Myocardial Fibers and Angiogenesis

Cardiac fibrosis is the main pathological feature of MI, and fibrosis is usually caused by excessive accumulation of extracellular matrix. Myofibroblasts are the main source of extracellular matrix, and they express the high-contractile protein *α*-SMA [28, 29]. The immunofluorescence of *α*-SMA can be used to evaluate the degree of myocardial fibrosis. The results showed that compared with the model group, *α*-SMA in the XFC group and EX527 group was significantly decreased (*P* < 0.01). Compared with the XFC group, *α*-SMA in the EX527 group was significantly increased (*P* < 0.01) (Figure 8(a)). Angiogenesis plays an important role in the recovery process of MI. As a marker of endothelial cells, CD31 represents the change in capillary density [30]. Compared with the sham group, CD31 in the model group was significantly increased (*P* < 0.01). Compared with the model group, the CD31 in the XFC group and the EX527 group was significantly increased (*P* < 0.01). Compared with the XFC group, the CD31 in the EX527 group was significantly decreased (*P* < 0.01) (Figure 8(b)). cTnI is a common method and index for clinical diagnosis of MI. AMI is usually accompanied by an increase in cTnI [31]. Compared with the sham group, the proportion obligation as previously described of cTnI in the model group was significantly increased (*P* < 0.01). Compared with the model group, the proportion of cTnI in the XFC group and the EX527 group was significantly decreased (*P* < 0.01). Compared with the XFC group, the proportion of cTnI in the EX527 group was significantly increased (*P* < 0.01) (Figure 8(c)).

## 4. Discussion

Cardiac repair after MI is accomplished through a series of complex events. These events begin with inflammation that helps digest and removes damaged cells and extracellular matrix tissues, followed by a repair phase with inflammation subsiding, fibroblast proliferation, scarring, and new angiogenesis in the following days [32]. Herbal formula contains hundreds of chemical compounds, which makes it complicated and challenging to understand the mechanisms of action and bioactive ingredients. Network pharmacology integrates data, and carries out experimental and clinical studies to provide a powerful tool for exploring the mechanisms of TCM [33]. In this work, we integrated network pharmacology, molecular docking, and experimental verification methods to clarify the molecular biological mechanism of XFC in the treatment of MI.

In this study, we first identified the active ingredients and targets of action of XFC, while obtaining disease targets for MI. We found that quercetin, kaempferol, *β*-sitosterol, luteolin, baicalein, stigmasterol, naringenin, and isorhamnetin were likely to be the main active ingredients of XFC to exert anti-MI. Most of these active ingredients are flavonoids; flavonoids can improve CVD, such as reducing the brittleness of blood vessels, improving the permeability of blood vessels, reducing lipids and cholesterol, and preventing hypertension [34–36]. For example, Albadrani et al. found that quercetin ameliorates MI in rats by decreasing TGF-*β*1/Smad3 signaling [37]. Wang et al. demonstrated that kaempferol ameliorates oxidative stress and inflammation by activating the PI3K/Akt/GSK-3*β* pathway, thereby reducing myocardial ischemia/reperfusion injury [38]. We next performed a PPI analysis on 147 overlapping targets to obtain the key targets among them. These key targets are mainly involved in apoptosis (TP53 and CASP3), immune inflammation (TNF, IL6), and angiogenesis (VEGFA), which are closely related to the molecular mechanisms of MI. MI evokes activation of the innate immune system, resulting in increased levels of proinflammatory cytokines (IL-1*β*, IL6, and TNF-*α*) in the heart and circulation. The TNF-mediated process is complex. TNF can show toxicity through TNFR1 and protection through TNFR2, showing bidirectional effects in MI [39]. VEGFA is a highly specific vascular endothelial growth factor that promotes angiogenesis and increases vascular permeability. VEGFA plays a key role in triggering the cardiac angiogenic response following MI. VEGFA can inhibit cardiomyocyte apoptosis, promote cardiac repair, and promote vasodilation [40, 41].

Combining our previous study and this bioinformatics analysis, we chose SIRT1 as an entry point among these key targets. First, we molecularly docked SIRT1 to the main active ingredients and found that SIRT1 can and stably bind, which confirmed that SIRT1 might be one of the targets of XFC. Then, we verified our hypothesis through experiments. Our data suggested that XFC can effectively improve cardiac function, myocardial fibrosis, and cardiomyocyte apoptosis in MI model rats. Interestingly, SIRT1 inhibitors could inhibit the effects of XFC, which confirms that SIRT1 may be the target of XFC. SIRT1, an NAD+-dependent protein deacetylase, is capable of deacetylating histones and nonhistone substrates that have a powerful regulatory role and can regulate a variety of important physiological and pathological processes in cells, such as cell metabolism, gene repair, cell survival, cell senescence, apoptosis, inflammatory response, oxidative stress, and vascular protection [42]. Previous studies have confirmed that activation of SIRT1 can alleviate MI injury [42, 43]. Based on this, we hypothesized that the active component of XFC could activate SIRT1 to exert its anti-MI effect.

The effect of promoting blood circulation and eliminating blood stasis in Chinese medicine is similar to that of angiogenesis. Recanalization and angiogenesis in the infarcted region are essential for the survival of cells in the myocardium. CD31 is an endothelial cell-specific marker that can be used to label vascular endothelial cells. *α*-SMA is a eukaryotic skeletal protein involved in the composition of microfilaments and is a marker protein for mesenchymal cells [44–46]. Our data suggest that XFC improved the expression of CD31 and *α*-SMA and that SIRT1 inhibitors eliminate this effect, so we hypothesize that XFC can exert a neovascularizing effect through SIRT1. Indeed, SIRT1 has been shown to improve CD31 and a-SMA expression, and this evidence further supports the reliability of our conclusions [47, 48].

## 5. Conclusion

In summary, we predicted by network pharmacology that SIRT1 might be a target of XFC against MI. The *in vivo* study showed that XFC could inhibit apoptosis, promote angiogenesis and improve myocardial fibrosis through SIRT1.

## Figures and Tables

**Figure 1:** Flow chart of this study.

**Figure 2:** Targets of XFC against MI: (a) overlapping targets of XFC against MI; (b) ingredients -target network.

**Figure 3:** PPI network of overlapping targets.

**Figure 4:** Gene enrichment analysis of overlapping targets: (a) KEGG enrichment analysis; (b) CC enrichment analysis; (c) BP enrichment analysis; (d) MF enrichment analysis.

**Figure 5:** Molecular docking of SIRT1 with major active ingredients.

**Figure 6:** The change in cardiac function in each group. ^##^*P* < 0.01 vs the sham group; ^*∗∗*^*P* < 0.01 vs the model group; ^△△^*P* < 0.01 vs the XFC group; *n* = 10.

**Figure 7:** The change of myocardial ischemia area in each group. (a) HE staining of heart tissue. (b) TUNEL images of cardiomyocytes; ^##^*P* < 0.01 vs the sham group; ^*∗∗*^*P* < 0.01 vs the model group; ^△△^*P* < 0.01 vs the XFC group; *n* = 10.

**Figure 8:** The change of *α*-SMA, CD31, and cTnI in the infarcted area in each group: (a) *α*-SMA; (b) CD31; (c) cTnI. ^##^*P* < 0.01 vs the sham group; ^*∗∗*^*P* < 0.01 vs the model group; ^△^*P* < 0.05, ^△△^*P* < 0.01 vs the XFC group; *n* = 10.

**Table 1:** The top 20 active ingredients of XFC.

Nos.	MOID	Names	Degree
1	MOL000098	Quercetin	364
2	MOL000422	Kaempferol	163
3	MOL000358	Beta-sitosterol	106
4	MOL000006	Luteolin	78
5	MOL002714	Baicalein	63
6	MOL000449	Stigmasterol	56
7	MOL004328	Naringenin	41
8	MOL000354	Isorhamnetin	30
9	MOL000173	Wogonin	26
10	MOL005828	Nobiletin	23
11	MOL002565	Medicarpin	20
12	MOL000392	Formononetin	19
13	MOL003896	7-methoxy-2-methyl isoflavone	19
14	MOL000497	Licochalcone a	18
15	MOL004891	Shinpterocarpin	18
16	MOL002773	Beta-carotene	17
17	MOL000500	Vestitol	16
18	MOL001689	Acacetin	15
19	MOL005003	Licoagrocarpin	15
20	MOL004957	HMO	15

## Data Availability

All data used to support the findings of this study are available from the corresponding author upon request.

## References

[1] Reed G. W., Rossi J. E., Cannon C. P. (Jan. 2017). Acute myocardial infarction. *The Lancet*.

[2] Anderson J. L., Morrow D. A. (2017). Acute myocardial infarction. *New England Journal of Medicine*.

[3] Hausenloy D. J., Yellon D. M. (2013). Myocardial ischemia-reperfusion injury: a neglected therapeutic target. *Journal of Clinical Investigation*.

[4] Heusch G. (2020). Myocardial ischaemia-reperfusion injury and cardioprotection in perspective. *Nature Reviews Cardiology*.

[5] Lin J., Wang Q., Hua X., Duan J., Yao K. (2022). Integrated gut-heart Axis and network pharmacology to reveal the mechanisms of the huoxue wentong formula against myocardial ischemia. *Evidence-based Complementary and Alternative Medicine*.

[6] Lin J., Wang Q., Zhou S., Xu S., Yao K. (2022). Tetramethylpyrazine: a review on its mechanisms and functions. *Biomedicine & Pharmacotherapy*.

[7] Liu T., Wang Q., Yao K. (2020). Huoxue Wentong Formula ameliorates myocardial infarction in rats through inhibiting CaMKII oxidation and phosphorylation. *Chinese Medicine*.

[8] Li Y., Tao T., Song D., He T., Liu X. (2021). Effects of xuefu zhuyu granules on patients with stable coronary heart disease: a double-blind, randomized, and placebo-controlled study. *Oxidative Medicine and Cellular Longevity*.

[9] Wang J., Yang X., Chu F. (2013). The effects of xuefu zhuyu and shengmai on the evolution of syndromes and inflammatory markers in patients with unstable angina pectoris after percutaneous coronary intervention: a randomised controlled clinical trial. *Evid Based Complement Alternat Med*.

[10] Zhang S., Chen Z.-L., Tang Y.-P., Duan J.-L., Yao K.-W. (2021). Efficacy and safety of xue-fu-zhu-yu decoction for patients with coronary heart disease: a systematic review and meta-analysis. *Evidence-based Complementary and Alternative Medicine*.

[11] Chang X., Zhang T., Meng Q. (2021). Quercetin improves cardiomyocyte vulnerability to hypoxia by regulating SIRT1/TMBIM6-related mitophagy and endoplasmic reticulum stress. *Oxidative Medicine and Cellular Longevity*.

[12] Chen M.-Q., Yao K.-W., Liu Z.-J., Feng X.-X., Xiao Y. (2020). Xuefu zhuyu oral liquid prevents apoptosis of ischemic myocardium cells in rats by regulating SIRT1 and its pathway-related genes. *Chinese Journal of Integrative Medicine*.

[13] Hopkins A. L. (2008). Network pharmacology: the next paradigm in drug discovery. *Nature Chemical Biology*.

[14] Li S., Zhang B. (2014). Traditional Chinese medicine network pharmacology: theory, methodology and application. *Chinese Journal of Natural Medicines*.

[15] Ru J., Li P., Wang J. (2014). TCMSP: a database of systems pharmacology for drug discovery from herbal medicines. *Journal of Cheminformatics*.

[16] Stelzer G., Rosen N., Plaschkes I. (2016). The GeneCards suite: from gene data mining to disease genome sequence analyses. *Current Protocols in Bioinformatics*.

[17] Piñero J., Ramírez-Anguita J. M., Saüch-Pitarch J. (2020). The DisGeNET knowledge platform for disease genomics: 2019 update. *Nucleic Acids Research*.

[18] Szklarczyk D., Gable A. L., Lyon D. (2019). STRING v11: protein-protein association networks with increased coverage, supporting functional discovery in genome-wide experimental datasets. *Nucleic Acids Research*.

[19] Shannon P., Markiel A., Ozier O. (2003). Cytoscape: a software environment for integrated models of biomolecular interaction networks. *Genome Research*.

[20] Zhou Y., Zhou B., Pache L. (2019). Metascape provides a biologist-oriented resource for the analysis of systems-level datasets. *Nature Communications*.

[21] Li J., Miao B., Wang S. (2022). Hiplot: a comprehensive and easy-to-use web service for boosting publication-ready biomedical data visualization. *Briefings in Bioinformatics*.

[22] Trott O., Olson A. J. (2010). AutoDock Vina: improving the speed and accuracy of docking with a new scoring function, efficient optimization, and multithreading. *Journal of Computational Chemistry*.

[23] Adasme M. F., Linnemann K. L., Bolz S. N. (2021). Plip 2021: expanding the scope of the protein-ligand interaction profiler to DNA and RNA. *Nucleic Acids Research*.

[24] Gomes K. M. S., Campos J. C., Bechara L. R. G. (Sep. 2014). Aldehyde dehydrogenase 2 activation in heart failure restores mitochondrial function and improves ventricular function and remodelling. *Cardiovascular Research*.

[25] Qin C., Zhang L., Wei H. (2010). *Laboratory Animal*.

[26] Wu Y., Xia Z.-Y., Zhao B. (2017). (−)-Epigallocatechin-3-gallate attenuates myocardial injury induced by ischemia/reperfusion in diabetic rats and in H9c2 cells under hyperglycemic conditions. *International Journal of Molecular Medicine*.

[27] Teng F., Li G., Liu Z., Zhang L., Yao K. (2014). The comparative study on expression of SIRT1 signal transduction by xuefuzhuyu Capsule. *Evid Based Complement Alternat Med*.

[28] Zeng Z., Wang Q., Yang X. (2019). Qishen granule attenuates cardiac fibrosis by regulating TGF-*β*/Smad3 and GSK-3*β* pathway. *Phytomedicine*.

[29] Jia D., Jiang H., Weng X. (2019). Interleukin-35 promotes macrophage survival and improves wound healing after myocardial infarction in mice. *Circulation Research*.

[30] Jin L., Pan Y., Li Q., Li J., Wang Z. (2021). Elabela gene therapy promotes angiogenesis after myocardial infarction. *Journal of Cellular and Molecular Medicine*.

[31] Liu J., Ning L. (2021). Protective role of emodin in rats with post-myocardial infarction heart failure and influence on extracellular signal-regulated kinase pathway. *Bioengineered*.

[32] Prabhu S. D., Frangogiannis N. G. (2016). The biological basis for cardiac repair after myocardial infarction: from inflammation to fibrosis. *Circulation Research*.

[33] Lai X., Wang X., Hu Y., Su S., Li W., Li S. (2020). Editorial: network pharmacology and traditional medicine. *Frontiers in Pharmacology*.

[34] Yu H., Chen B., Ren Q. (2019). Baicalin relieves hypoxia-aroused H9c2 cell apoptosis by activating Nrf2/HO-1-mediated HIF1*α*/BNIP3 pathway. *Artificial Cells, Nanomedicine, and Biotechnology*.

[35] Dehghani F., Sezavar Seyedi Jandaghi S. H., Janani L., Sarebanhassanabadi M., Emamat H., Vafa M. (2021). Effects of quercetin supplementation on inflammatory factors and quality of life in post-myocardial infarction patients: a double blind, placebo-controlled, randomized clinical trial. *Phytotherapy Research*.

[36] Micek A., Godos J., Del Rio D., Galvano F., Grosso G. (2021). Dietary flavonoids and cardiovascular disease: a comprehensive dose-responsemeta-analysis. *Molecular Nutrition & Food Research*.

[37] Albadrani G. M., BinMowyna M. N., Bin-Jumah M. N., El–Akabawy G., Aldera H., Al A. M. (2021). Quercetin prevents myocardial infarction adverse remodeling in rats by attenuating TGF-*β*1/Smad3 signaling: different mechanisms of action. *Saudi Journal of Biological Sciences*.

[38] Wang D., Zhang X., Li D. (2017). Kaempferide protects against myocardial ischemia/reperfusion injury through activation of the PI3K/Akt/GSK-3*β* pathway. *Mediators of Inflammation*.

[39] Gouweleeuw L., Wajant H., Maier O., Eisel U., Blankesteijn W., Schoemaker R. (2021). Effects of selective TNFR1 inhibition or TNFR2 stimulation, compared to non-selective TNF inhibition, on (neuro)inflammation and behavior after myocardial infarction in male mice. *Brain, Behavior, and Immunity*.

[40] Tao Z., Chen B., Tan X. (2011). Coexpression of VEGF and angiopoietin-1 promotes angiogenesis and cardiomyocyte proliferation reduces apoptosis in porcine myocardial infarction (MI) heart. *Proceedings of the National Academy of Sciences of the United States of America*.

[41] Braile M., Marcella S., Cristinziano L. (2020). VEGF-A in cardiomyocytes and heart diseases. *International Journal of Molecular Sciences*.

[42] D’Onofrio N., Servillo L., Balestrieri M. L. (2018). SIRT1 and SIRT6 signaling pathways in cardiovascular disease protection. *Antioxidants and Redox Signaling*.

[43] Wang L.-Z., Xi J.-N., Liu T.-J., Zhang Z.-Y., Zhang P. (2020). MiR-204 reduces apoptosis in rats with myocardial infarction by targeting SIRT1/p53 signaling pathway. *European Review for Medical and Pharmacological Sciences*.

[44] Zeisberg E. M., Kalluri R. (2010). Origins of cardiac fibroblasts. *Circulation Research*.

[45] Makarevich P. I., Dergilev K. V., Tsokolaeva Z. I. (May 2018). Angiogenic and pleiotropic effects of VEGF165 and HGF combined gene therapy in a rat model of myocardial infarction. *PLoS One*.

[46] Pang J., Ye L., Chen Q. (2020). The effect of MicroRNA-101 on angiogenesis of human umbilical vein endothelial cells during hypoxia and in mice with myocardial infarction. *BioMed Research International*.

[47] Liu Z.-H., Zhang Y., Wang X. (2019). SIRT1 activation attenuates cardiac fibrosis by endothelial-to-mesenchymal transition. *Biomedicine & Pharmacotherapy*.

[48] Wang Y., Zuo B., Wang N., Li S., Liu C., Sun D. (2020). Calcium dobesilate mediates renal interstitial fibrosis and delay renal peritubular capillary loss through Sirt1/p53 signaling pathway. *Biomedicine & Pharmacotherapy*.

